# The Comparison of the Diagnostic Value of Left Atrial Pulmonary Vein Single-Phase and Dual-Phase Enhanced CT Scanning for Left Atrial Appendage Thrombosis and SEC in Patients with Atrial Fibrillation

**DOI:** 10.1155/2022/8679511

**Published:** 2022-05-14

**Authors:** Tianjiao Guo, Yapeng Dong, Shujing Yu

**Affiliations:** Department of Radiology, Cangzhou Central Hospital, Hebei Medical University, Cangzhou, Hebei 061001, China

## Abstract

**Objective:**

The accuracy of left atrial pulmonary vein CT enhanced single-phase and dual-phase scanning in the detection of left atrial appendage (LAA) thrombosis and spontaneous echo contrast (SEC) before radio frequency ablation was compared in atrial fibrillation patients, so as to optimize the scanning scheme.

**Methods:**

78 patients with atrial fibrillation who were admitted to Cangzhou Central Hospital from October 2020 to September 2021 and underwent bilateral enhanced CT scan of left atrial pulmonary vein and transesophageal echocardiography (TEE) examination for planned frequency ablation were selected. TEE results were used as the “gold standard” to compare the diagnostic efficacy of the first phase, second phase, and double-phase comprehensive mode of enhanced left atrial pulmonary vein CT in detecting left atrial thrombosis and SEC.

**Results:**

The sensitivity, specificity, positive predictive value, and negative predictive value were 88.9%, 84.1%, 42.1%, and 98.3%, respectively, in the detection of left atrial thrombosis and SEC by the first phase of CT enhanced scan. The sensitivity, specificity, positive predictive value, and negative predictive value were 22.2%, 98.6%, 66.6%, and 90.7%, respectively, in the detection of left atrial thrombosis and SEC by the second phase of CT enhanced scan. The sensitivity, specificity, positive predictive value, and negative predictive value were 88.9%, 84.1%, 42.1%, and 98.3%, respectively, in the detection of left atrial thrombosis and SEC by the double-phase comprehensive mode of CT enhanced scan. There was no statistically significant difference in the accuracy of CT diagnosis of left atrial appendage thrombosis and SEC between the three modes of the first phase, the second phase, and the double-phase comprehensive CT (*P* > 0.05). The mean effective radiation dose of double-phase enhanced scan was 7.49 ± 1.02 mSv.

**Conclusion:**

Single-phase enhanced CT scan of left atrial pulmonary vein can meet clinical requirements and significantly reduce the radiation dose compared with double-phase enhanced CT scan. Therefore, it is recommended as an initial screening examination for patients with atrial fibrillation before radiofrequency ablation.

## 1. Introduction

Atrial fibrillation (AF) is one of the most common arrhythmias in clinic and has attracted much clinical attention because it can cause serious thromboembolic events. Currently, pulmonary vein antrum isolation (PVAI) and other radiofrequency ablation have gradually become the main measures for clinical treatment of atrial fibrillation, while left auricular thrombosis is an absolute contraindication in PVAI [1]. It has been found that SEC represents blood stasis and prethrombotic state and is associated with an increasing risk of thromboembolism in patients with NVAF [2–4]. Gedikli et al.'s [5] analysis found that patients with dense SEC had a 3.7-fold increased risk of stroke. Anticoagulant therapy should also be performed for patients with SEC in LAA [6]. Left atrial appendage closure (LAAC) can be performed for patients with contraindication or rejection of anticoagulant therapy [7]. Wang et al. [8] found that left atrial appendage closure was safe and effective in NVAF patients with SEC. Therefore, it is of equal clinical significance for atrial fibrillation patients to identify left atrial appendage thrombosis and SEC before PVAI. Transesophageal echocardiography is the gold standard for the examination of LAA thrombosis and SEC. However, TEE currently has many shortcomings, such as many contraindications and painful examination, which may cause esophageal injury, severe arrhythmia, myocardial infarction, and other serious complications. The accuracy of the examination results mainly depends on the experience of the operator, and TEE cannot accurately evaluate the anatomical relationship between pulmonary vein and left atrium, and the spatial anatomical structure is not good, due to the poor repeatability of invasive examination [9]. Left atrial pulmonary vein enhancement CT scan as a noninvasive imaging technology, can objectively and stereoscopically display anatomical relation between the left atrium and pulmonary veins and anatomical structure, prompts variation situation of pulmonary vein, can carry on the standard measuring accurately along the pulmonary vein, and enables the radiofrequency ablation surgery to be personal according to the patient's anatomical variations and individualization. Contrast-enhanced CT scanning of left atrial pulmonary vein has been widely recognized clinically [10, 11], and studies have proved that contrast-enhanced CT has great application value in the detection of LAA thrombus and SEC [12, 13]. In this study, TEE results were used as the “gold standard” to evaluate the diagnostic efficacy and clinical significance of the first phase, the second phase, and the double-phase comprehensive enhanced CT of the left atrial pulmonary vein for left atrial thrombosis and SEC in patients with atrial fibrillation, so as to optimize the scanning scheme.

## 2. Data and Methods

### 2.1. The General Data

A total of 81 patients with atrial fibrillation who were admitted to Cangzhou Central Hospital from October 2020 to September 2021 and underwent bilateral enhanced CT scan of left atrial pulmonary vein and transesophageal echocardiography (TEE) examination were selected. (1) The interval between enhanced CT scan and TEE was more than 2 days; (2) CT image quality is poor and affects assessment; (3) accompanied by heart disease that affects the test results; and (4) esophageal varices, strictures, malformations, and other esophageal diseases that affect the examination results. A total of 78 patients were included, including 28 females (35.9%) and 50 males (64.1%), aged from 26 to 79 years, with an average age of 52.5 ± 26.5 years. All 78 patients were diagnosed with paroxysmal atrial fibrillation. Duration of illness is 6 months to 5 years. All patients signed informed consent prior to examination.

### 2.2. Examination Method

#### 2.2.1. Left Atrial Pulmonary Vein Enhanced CT Scan

Toshiba Aquilion One 320-row dynamic volume CT was used for scanning. Supine position was adopted with feet advanced, arms were raised above the head, cardiac conductance was connected, and the scanning was carried out at the end of a single inhalation. According to the anteroposterior-lateral positioning images, the scanning range was determined from the tracheal carina to the diaphragmatic surface of the heart, with a range of about 140-160 mm, covering the whole heart.

The nonionic contrast agent iohexol 350 60-65 mL was injected through the elbow vein at a rate of 4.5-5.0 mL/s with a Mallinckrodt double-cavity high-pressure syringe. The flow rate was adjusted according to the patient's BMI and vascular condition, and then, 40 mL of normal saline was injected at the same rate. The monitoring was started 10 s after the injection of contrast agent, and the left ventricle was selected as the monitoring area for manual triggering, with the trigger threshold of 150 HU. The second scanning interval is 6 s. Scanning parameters were as follows: tube voltage 120 kV and current adopts automatic modulation mode. The scanning layer thickness and spacing were 0.5 mm, the rotation speed was 0.35 s/lap, and the average scanning time was 12-15 s. After scanning, the optimal phase reconstruction was selected and sent to AW4.6 workstation. Based on the cross-sectional image, multiplane reconstruction (MPR), maximum intensity projection (MIP), volume reproduction (VR), and other reconstruction methods were used to reconstruct the image. The CT examination results were concluded by the joint study of two experienced CT diagnostic physicians. If the two doctors have different opinions on the results, the chief physician shall be invited to participate in the discussion and the final results will be obtained.

The evaluation criteria of CT results were as follows:(1) the contrast agent in the LAA of the first and second scans was completely filled, and the diagnosis was negative. (2) The first phase of LAA showed a local filling defect with contrast agent, while the second phase of LAA was not filled with contrast agent. At the same time, the image differentiated from the comb muscle was diagnosed as thrombus. Filling defect at any phase is positive. LAA filling defect in the first phase, contrast agent filling in the second phase, or LAA is completely filled in the first phase of contrast agent, and filling defect occurs in the second phase of LAA, which is SEC phenomenon. In the measurement of anterior and posterior diameters of the left atrium, the left atrium is relatively less affected by heartbeat, and the maximum cross-section of the left atrium is usually at the level of the right lower pulmonary vein. Mediastinal CT images (window width 350 HU, window location 40 HU) were used for measurement, and the anterior and posterior diameters of the left atrium were measured under this condition [14].

#### 2.2.2. TEE Examination

Philips iE33 ultrasound system was used in all patients for ultrasonic diagnosis, with a probe of 2.0~7.0 MHZ. The transesophageal ultrasound probe was placed in the esophagus, 30~40 cm away from the incisors. During the inspection, LAA was continuously scanned at 0~180° from multiple angles and different depths to clearly display its shape and internal structure. The result of TEE examination was concluded by the joint study of two experienced sonographers. If the two doctors have different opinions on the result, the chief doctor will be invited to participate in the discussion and the final result will be obtained.

TEE was found to be positive: (1) SEC: cloud-like echo of cyclotron movement in left atrium or left atrial appendage and unrelated to cardiac cycle. When noise artifact was excluded, SEC was diagnosed. (2) Thrombus: old thrombus is a mass tissue with clear boundary, different ultrasonic echoes from surrounding myocardium, and independent degree of activity and can be observed at two vertical angles [15]; fresh thrombus: if the observed mass is deformable and active by TEE, part of it can be flushed by the blood flow of LAA with the change of cardiac cycle; then, it is considered as fresh thrombus.

### 2.3. Statistical Analysis

SPSS19.0 statistical software was used for data analysis. Measurement data were expressed as mean ± standard deviation, and *t* test was used for homogeneity of variance and normal distribution. When *P* < 0.05, the difference was statistically significant. TEE was used as the standard to evaluate the sensitivity, specificity, positive predictive value, and negative predictive value of the first, second, and double-phase comprehensive diagnosis of thrombus and SEC in LAA.

## 3. Results

Among the 78 patients with atrial fibrillation who underwent enhanced CT scanning of left atrial pulmonary vein, 19 patients with filling defect in LAA were found by CT scanning of the first phase, 3 patients were diagnosed as having thrombosis by TEE, 5 patients were diagnosed as having SEC, and 11 patients were negative. A total of 3 cases were found to be positive by the second-phase CT, 2 cases were diagnosed as having thrombosis by TEE, and 1 case was negative. A total of 19 patients were diagnosed as positive by double-phase comprehensive CT (3 cases were thrombosis, 16 cases of SEC), among which 2 cases of thrombosis were confirmed by TEE, and 1 case was negative. Five cases of SEC were confirmed by TEE, 1 case of fresh thrombosis was confirmed, and 10 cases were negative. There were 59 patients with negative CT diagnosis at the first phase, 1 patient was confirmed as having thrombosis by TEE, and the rest were normal. The second CT diagnosis was negative in 75 cases, 5 cases were diagnosed as having SEC by TEE, 2 cases were diagnosed as having thrombosis, and the rest were normal. There were 59 negative patients diagnosed by double-phase comprehensive CT, 1 patient was diagnosed as having thrombosis by TEE, and the rest were normal (Figures 1–3). There was no statistically significant difference in the comparison of the prediction accuracy of the first phase, the second phase, and the double-phase comprehensive in CT scanning (*P* > 0.05) (Table 1). Using TEE results as the “gold standard,” the sensitivity, specificity, positive predictive value, and negative predictive value of the first CT scan in the diagnosis of left atrial fibrillation and SEC were 88.9%, 84.1%, 42.1%, and 98.3%, respectively. The sensitivity, specificity, positive predictive value, and negative predictive value of the second CT scan in the diagnosis of left atrial fibrillation and SEC were 22.2%, 98.6%, 66.6%, and 90.7%, respectively. The sensitivity, specificity, positive predictive value, and negative predictive value of double-phase comprehensive CT in the diagnosis of left atrial fibrillation and SEC were 88.9%, 84.1%, 42.1%, and 98.3%, respectively (Table 2). In this study, CT scan results were negative in the first phase and 0 positive patient in the second phase. In 78 patients, 1 patient was missed by the first phase and double-phase scanning.

The anterior and posterior diameter of the left atrium was 44.9 ± 15.5 mm.

The mean double-phase effective radiation dose of pulmonary vein enhancement was 7.49 ± 1.02 mSv.

## 4. Discussion

The purpose of this study was to combine LAA thrombosis and SEC as positive indicators requiring intervention and compare the value of single-phase and dual-phase scanning, so as to optimize the scanning program and provide a safe and reliable preoperative evaluation method for patients with atrial fibrillation undergoing radiofrequency ablation.

SEC phenomenon first appeared in ultrasound imaging. In patients with atrial fibrillation, due to irregular atrial contraction, the left atrium and left atrial appendage have different degrees of structural remodeling, myocardial cell hypertrophy, decreased vitality, and decreased or even disappeared muscle fibers. And glycogen storage in mitochondria reduces its activity and further results in the decrease of myocardial contraction force; LAA blood flow is slow, smaller shear stress superposition of red blood cells, ultrasonic gathered in a fold together in the backward scattering field of the red blood cells, to produce a mist sex during ultrasound through echo, the phenomenon of the SEC [4]. The average anterior-posterior diameter of the left atrium in the 78 patients in this group was 44.9 mm, significantly larger than the normal value, reflecting the structural changes of the left atrium in patients with atrial fibrillation, which was consistent with the above theory.

We defined the SEC phenomenon on CT as LAA filling defect in the first phase and contrast agent filling in the second phase or LAA filling defect in the second phase and contrast agent filling in the first phase. However, there was no single second-phase filling defect in the 78 patients in this group, which may be due to the different imaging principles of CT and TEE. SEC is only blood stasis [12], and the filling and excretion of contrast agent are slow. Once filled, it is difficult to discharge in a very short time, so there will not be a single second-phase filling defect. SEC often occurs in LAA, because the left atrial appendage has a complex shape, which is spiral with large curvature, and there are abundant comb muscles and trabecular muscle, which easily causes hemodynamic disorder in the left atrial appendage, reduce blood flow velocity in LAA, and prolong the filling and excretion time of contrast agent [16–18].

The CT examination method of the patients in this group was double-phase enhanced CT scan of left atrial pulmonary vein. From the perspective of the consistency of CT results with TEE, there was no statistically significant difference in the comprehensive prediction of the first, second, and double phase (*P* = 0.560), which was considered to be related to the majority of negative cases in this group. Using TEE results as the “gold standard,” the sensitivity, specificity, positive predictive value, and negative predictive value of LAA thrombosis and SEC were 88.9%, 84.1%, 42.1%, and 98.3%; 22.2%, 98.6%, 66.6%, and 90.7%; and 88.9%, 84.1%, 42.1%, and 98.3% in the first, second, and double-phase comprehensive evaluation, respectively. The sensitivity of the second-phase CT scan in the diagnosis of left atrial appendage thrombosis and SEC was 22.2%, which was significantly lower than that of the first phase, and 4 cases of missed diagnosis of thrombosis were 2 cases. All 5 cases of SEC were missed. Its value lies in the initial distinction between thrombus and SEC in conjunction with the first phase scans. Since no new filling defect was found in the second phase, the sensitivity, specificity, positive predictive value, and negative predictive value of the first and second phase comprehensive diagnosis of thrombi and SEC in LAA were the same. Therefore, based on the purpose of detecting LAA thrombus and SEC, the value of the first phase scanning was significantly higher than that of the second phase scanning, which was equivalent to double-phase comprehensive. The first phase scan had a high sensitivity (88.9%) for the diagnosis of thrombosis and SEC and a high negative predictive value (98.3%). It is suggested that LAA thrombosis and SEC can be basically excluded when CT examination results are negative, especially for patients with contraindications to TEE examination; it can be used as an alternative examination of TEE. However, due to the high false-positive rate of SEC in the first phase of scan diagnosis (11 cases), TEE examination is still needed to confirm the diagnosis of patients with positive CT results.

There are many studies on the diagnosis of left atrial internal thrombosis by multiphase scanning or changing the delay time of dual-phase scanning, which undoubtedly increases the radiation dose of patients. At present, there is a lack of unified standards for left atrial pulmonary vein enhanced CT scanning protocols, including single-phase, dual-phase, and multiphase scanning protocols [12, 19, 20]. Double-phase scanning was used in this study, and the average effective radiation dose of patients was 7.49 ± 1.02 mSv. With the deepening of people's understanding of SEC, the value of using CT to distinguish thrombi from SEC gradually decreases. The reduction of radiation dose has become a major concern. The results showed that single-phase enhanced CT scan of left atrial pulmonary vein could obtain the highest diagnostic efficiency and significantly reduce the radiation dose.

In a word, left atrial pulmonary vein single-phase enhanced CT scan as a noninvasive examination method, the accurate assessment of pulmonary vein at the same time, the LAA thrombosis, and the SEC, has high sensitivity and high negative predictive value and can meet the demand of radiofrequency ablation of atrial fibrillation patients before evaluation but also significantly reduce the radiation dose compared with the double-phase enhanced scan. It is recommended as an initial screening test for patients with atrial fibrillation before radiofrequency ablation.

## Figures and Tables

**Figure 1:** A 68-year-old woman with atrial fibrillation. (a) TEE showed a hyperechoic mass with a size of 11.8 mm × 9.2 mm in the middle part of left atrial appendage (arrow); (b, c) are CT images of the first phase and the second phase. No filling defect area corresponding to thrombus was found in LAA on CT images. The arrow in (c) refers to the pecinate muscles with a diameter of about 4.77 mm.

**Figure 2:** A 56-year-old male with atrial fibrillation. (a) TEE showed foggy changes in the left atrium and left atrial appendage (arrow); (b) left atrial pulmonary vein double-phase enhanced CT scan showed the filling defect area with unclear boundary in the first phase of LAA (arrow), and the filling defect area was uniformly filled with contrast agent in the second phase of (c) (arrow).

**Figure 3:** A 74-year-old male with atrial fibrillation. (a) TEE showed a foggy change in the left atrium and a hyperechoic mass of 18.2 × 8.1 mm in the middle and lower segment of the left atrial appendage (arrow). (b) Left atrial pulmonary vein double-phase enhanced CT scan showed clear boundary filling defect (arrow) in the first phase of LAA, while the filling defect area in the second phase of (c) showed no significant change (arrow).

**Table 1:** Comparison of comprehensive prediction of left atrial pulmonary vein enhanced CT in the first phase, the second phase, and double-phase comprehensive.

	Same	Different	*X* ^2^ value	*P* value
First-phase CT	66 (84.6%)	12 (15.4%)	1.158	0.560
Second-phase CT	70 (89.7%)	8 (10.3%)		
Double-phase CT	66 (84.6%)	12 (15.4%)		

**Table 2:** The diagnostic efficacy of left atrial pulmonary vein enhanced CT in different periods for thrombosis and SEC.

Group	Sensitivity	Specificity	Positive predictive value	Negative predictive value
The first phase	88.9%	84.1%	42.1%	98.3%
The second phase	22.2%	98.6%	66.7%	90.7%
The double phase	88.9%	84.1%	42.1%	98.3%

## Data Availability

The simulation experiment data used to support the findings of this study are available from the corresponding author upon request.
